The article "Knockdown of PVT1 Exerts Neuroprotective Effects against Ischemic Stroke Injury through Regulation of miR-214/Gpx1 Axis" was retracted in 2023. Reasons: suspected computer-generated content; unreliable results or conclusions; concerns about the data; concerns about the results or conclusions.

# Knockdown of PVT1 Exerts Neuroprotective Effects against Ischemic Stroke Injury through Regulation of miR-214/Gpx1 Axis

**DOI:** 10.1155/2022/1393177

**Published:** 2022-08-08

**Authors:** Xiaozhou Liu, Tian Wang, Ping Jing, Mei Zhang, Fei Chang, Wei Xiong

**Affiliations:** Department of Neurology, The Central Hospital of Wuhan, Tongji Medical College, Huazhong University of Science and Technology, Wuhan 430014, China

## Abstract

Previous studies have reported that lncRNA PVT1 was closely related to ischemic stroke. Here, the role of PVT1 in ischemic stroke and the underlying mechanism were investigated. OGDR-stimulated PC12 cells were used to construct a cell model to mimic ischemic stroke. si-PVT1, miR-214 mimic, inhibitor, or the negative controls were transfected into PC12 cells prior to OGDR treatment. PVT1, miR-214, and Gpx1 expression was measured by qRT-PCR and western blotting assays. Cell proliferation and apoptosis were tested by CCK-8 assay and western blotting. The expression levels of inflammatory factors were determined by ELISA Kit. Results showed that PVT1 was increased significantly in OGDR PC12 cells. PVT1 knockdown significantly enhanced cell viability and attenuated cell apoptosis, ROS generation, and inflammation in OGDR PC12 cells. More importantly, PVT1 or Gpx1 was a target of miR-214. Mechanistically, PVT1 acted as a competing endogenous RNA of miR-214 to regulate the downstream gene Gpx1. In conclusion, PVT1 knockdown attenuated OGDR PC12 cell injury by modulating miR-214/Gpx1 axis. These findings offer a potential novel strategy for ischemic stroke therapy.

## 1. Introduction

Ischemic stroke is the most common cause of disability and death among adults worldwide. The current clinical effective treatment is to restore blood flow as soon as possible. However, the short treatment time and the high risk of secondary damage limit the applicability. Ischemic stroke involves several pathophysiological mechanisms, such as inflammatory response, cytotoxicity, and oxidative stress-induced necrosis or neuronal apoptosis, which is rather complex. Therefore, finding new therapeutic targets is essential for the treatment of ischemic stroke.

Long noncoding RNA (lncRNA), an emerging regulatory RNA, regulates gene expression at posttranscriptional levels. Previous research has reported that lncRNAs play important regulatory roles in the physiological processes of multiple diseases including stroke, malignancies, chronic lung diseases, and cardiovascular diseases [1–3]. For instance, Wang et al. displayed that lncRNA MALAT1 was upregulated in ischemic stroke and MALAT1 knockdown facilitated cell viability and suppressed cell apoptosis [4]. Knockdown of SNHG15 protected against ischemic stroke injury via inhibiting neuronal apoptosis and suppressing infarct area [5]. Fan et al. discovered that inactivation of H19 inhibited the functional recovery in MCAO rats [6]. lncRNA plasmacytoma variant 1 (PVT1) has been considered a candidate oncogene in various cancers, including breast cancer, glioblastoma, and bladder cancer [7–9]. Liu et al. discovered that PVT1 was obviously increased in acute ischemic stroke patients, suggesting PVT1 might be a potential diagnostic biomarker. However, the role of PVT1 in ischemic stroke remains largely unclear.

MicroRNAs (miRNAs), short single-stranded RNAs, exert diverse functions in various pathological processes via regulating gene expression at posttranscriptional level [10–14]. Previous studies have reported that the dysregulation of miRNAs was related to ischemic stroke, such as miR-143, miR-190, miR-195, and miR-451 [15–17]. Lu et al. displayed that miR-214 was elevated in ischemia stroke patients, indicating the association of miR-214 with ischemic stroke. Thereby, miR-214 was speculated to be involved in the pathogenesis of ischemic stroke.

Glutathione peroxidase 1 (Gpx1) is an essential component of the intracellular antioxidant enzyme. Increasing evidence has demonstrated that Gpx1 exhibited a critical role in the progress of brain diseases. For instance, Gpx1 was found to be increased in glioma [18]. Sharma et al. found that Gpx1 silencing promoted the proinflammatory response and activated vascular endothelium [19]. Moreover, Karahalil et al. reported that Gpx1 served as a risk factor for ischemic stroke [20], indicating that Gpx1 might be involved in the development of ischemic stroke.

Long noncoding RNA (lncRNA) was another emerging regulatory RNA, interacting with miRNA through conserved sequences to release mRNAs from RNA-induced silencing complexes. Prior studies have shown that miR-214 served as a target of PVT1 in regulation of hepatocellular carcinoma, ovarian cancer, and diabetic cataract [21–23]. Here, we speculated whether lncRNA PVT1 modulated cerebral ischemic stroke through targeting miR-214. Xiao et al. discovered that Gpx1 was a target of miR-214 in acute lymphoblastic leukemia [2]. In this present study, we performed an OGDR model in PC12 cells to explore the role of PVT1 in ischemic stroke injury and its underlying mechanism involved.

## 2. Material and Methods

### 2.1. Cell Culture

PC12 cells were obtained from the Chinese Academy of Sciences (Shanghai, China). They were cultured in DMEM (Gibco, USA) containing with 10% FBS (Life Science, USA) at 37°C in a humidified incubator containing 5% CO_2_.

### 2.2. Establishment of OGDR Model

The model was constructed following the instructions described previously [24]. In brief, PC12 cells, purchased from Shanghai Institutes of Cell Biological Sciences (Shanghai, China), were exposed to OGD for 2 h at 37°C and then returned to a normal environment. PC12 cells were incubated in an anaerobic chamber with 95% N_2_ and 5% CO_2_ without glucose. Subsequently, the cells were transferred to a normoxic conditions for 24 h to reoxygenation. The sham group was performed with the same treatment except for OGD exposure.

### 2.3. Cell Transfection

PVT1 small interfering RNA (PVT1 siRNA), pcDNA-PVT1 overexpression vector (pcDNA-PVT1), Gpx1 plasmid vector (Gpx1 vector), and miR-214 mimic/inhibitor were designed and synthesized by GenePharma (Shanghai, China). With the help of Lipofectamine 2000 Reagent (Invitrogen, Carlsbad, USA), the transfections were performed for 24 h, according to the protocol company's instructions.

### 2.4. Quantitative Reverse Transcription-Polymerase Chain Reaction (qRT-PCR)

Total RNA was extracted using TRIzol reagent (Invitrogen; Thermo Fisher Scientific, Inc.). The TaqMan miRNA assays were applied to perform RT-qPCR reactions. The ABI PRISM 7700 sequence detection system (Thermo, Waltham, USA) was used to run all reactions. The relative expression was calculated using the 2-*ΔΔ*Ct method and was normalized to U6 or GAPDH.

### 2.5. MTT Assay

2 × 10^4^ PC12 cells were cultured for 24 h. MTT solution (5 mg/mL, Sigma) was added and incubated 4 h at 37°C. Afterwards, 150 *μ*L DMSO (Beijing, China) was added and incubated for 1 h. The absorbance at 490 nm was detected using a microplate reader (Bio-Tek, Winooski, USA).

### 2.6. Western Blotting Assay

50 *μ*g of samples isolated from PC12 cells was separated by SDS-PAGE, followed by transferred to PVDF membranes (Millipore, Billerica, MA, USA). Afterwards, the membranes were incubated with 5% BSA, the primary antibodies against Bax (Abcam, ab32503, 1 : 1000), Bcl-2 (Abcam, ab182858, 1 : 2000), cleaved-caspase-3 (Abcam, ab32042, 1 : 1000), pro-caspase-3 (Abcam, ab32150, 1 : 1000), Gpx1 (Abcam, ab22604, 1 : 1000), and GAPDH (Cell Signaling Technology, #97166, 1 : 1000) and the secondary HRP antibodies (Abcam, ab205718, ab205719, 1 : 2000). The bands were detected by an ECL detection system (Pierce, Rockford, USA), and the quantification was performed by Image Lab™ Software (Bio-Rad, Shanghai, China).

### 2.7. ELISA Assay

The ELISA kits (Sigma) purchased from Beyotime Biotechnology (Beijing, China) were applied to detect the activity of ROS and inflammatory cytokines in PC12 cells with different treatment. The microplate reader (Bio-Tek, Winooski, USA) was applied to measure the optical density of each group at 450 nm.

### 2.8. Luciferase Reporter Assay

PC12 cells were transfected together with miR-214 mimic and constructed pGL3 luciferase vector (Promega, Madison, USA) using Lipofectamine 2000 reagent (Invitrogen). 48 h after transfection, the relative luciferase activity was analyzed by the dual luciferase reporter assay system (Promega, Madison, USA) and normalized to Renilla luciferase activity.

### 2.9. RIP Assay

PC12 cells were lysed in RIP buffer containing magnetic beads conjugated with anti-Ago2 antibody, negative control IgG, and positive control Input. Cells were incubated with Proteinase K buffer, and the RNA was extracted by TRIzol regent after washed by ice-cold saline water (150 mmol/L NaCl), and the purified RNA expression were analyzed by qRT-PCR.

### 2.10. Statistical Analysis

The experimental data were expressed as the mean ± standard deviation (SD). The differences between two or more groups were analyzed using two-tailed Student's *t*-tests or one -way ANOVA followed by Turkey's post hoc test, respectively. Statistical analysis was performed using SPSS Statistics 20.0 software (IBM Corp.) and GraphPad Prism version 6.0 software (GraphPad Software Inc.). *p* < 0.05 was considered statistically significant.

## 3. Results

### 3.1. PVT1 and Gpx1 Were Increased, and miR-214 Was Decreased in an Ischemic Stroke Cell Model

To evaluate the levels of PVT1, miR-214, and Gpx1 affected by ischemia stroke, the OGDR model in PC12 cells was established. qRT-PCR results showed that PVT1 was overexpressed, while miR-214 was underexpressed in OGDR PC12 cells (Figures 1(a) and 1(b)). Results from western blotting discovered that Gpx1 level was highly expressed as well in OGDR PC12 cells (Figure 1(c)). These data indicated that OGD enhanced PVT1 and Gpx1 level, while inhibiting miR-214 level.

### 3.2. PVT1 Knockdown Promoted Cell Proliferation and Alleviated Apoptosis, ROS Generation, and Inflammation in Ischemic Stroke Cells

To evaluate the functional role of PVT1 on ischemic stroke, the loss of function experiments in OGDR PC12 cells were performed. As shown in Figure 2(a), PVT1 expression was obviously lower in si-PVT1 group than in the si-NC group. CCK-8 results indicated that PVT1 knockdown promoted cell viability reduced by OGDR operation (Figure 2(b)). Moreover, the PCNA expression was increased by si-PVT1, which was reduced by OGDR operation (Figure 2(c)). These findings indicated that PVT1 inhibition facilitated cell proliferation in ischemic stroke cells. In addition, western blotting results discovered that si-PVT1 inhibited Bcl-2 level, while enhancing Bax and cleaved-caspase-3 levels in OGDR PC12 cells (Figure 2(d)), indicating the inhibitory effect of si-PVT1 on OGDR PC12 cells apoptosis. Furthermore, the ROS generation and inflammatory cytokines in OGDR PC12 cells were increased significantly under OGDR operation, and knockdown of PVT1 obviously reduced these levels (Figures 2(e) and 2(f)). These findings indicated that PVT1 knockdown enhanced cell proliferation and alleviated apoptosis, ROS generation, and inflammation in ischemic stroke cells.

### 3.3. PVT1 Functions as a ceRNA of miR-214 in PC12 Cells

To explore the molecular mechanism of PVT1 in ischemic stroke, Starbase was first used to identify the miRNAs interacting with PVT1 in PC12 cells. The binding sites for miR-214 in PVT1 are shown in Figure 3(a). To further identify the interaction between miR-214 and PVT1, RIP and dual luciferase reporter assays were applied. Restoration of miR-214 obviously increased miR-214 expression, when compared with the control group (Figure 3(b)). Results from luciferase reporter assays found that PVT1-WT luciferase activity in PC12 cells was significantly decreased by miR-214 mimic; however, there was no change in the PVT1-MuT group (Figure 3(c)). Meanwhile, RIP results manifested that the levels of PVT1 and miR-214 were increased in the Ago2 group compared to the negative control IgG group. Compared with the Input group, the two groups of samples have good parallelism (Figure 3(d)). Moreover, PVT1 was significantly upregulated by treatment with pcDNA-PVT1 (Figure 3(e)). Furthermore, PVT1 knockdown enhanced cell viability and attenuated cell apoptosis, ROS generation, and inflammation in OGDR PC12 cells, while PVT1 overexpression inhibited miR-214 expression in PC12 cells (Figure 3(f)). These results demonstrated that PVT1 was directly binding to miR-214 in PC12 cells.

### 3.4. miR-214 Directly Targeted Gpx1

To observe the target of miR-214 in PC12 cells, TargetScan and miRDB were applied. As shown in Figure 4(a), miR-214 possessed very high binding affinities with Gpx1. Moreover, the luciferase activities in PC12 cell o-transfection of Gpx1-WT vector and miR-214 mimic were decreased remarkably compared with the Gpx1-MuT vector (Figure 4(b)). In addition, overexpression of miR-214 significantly inhibited Gpx1 expression, which is shown in Figures 4(c) and 4(d) by western blotting and RT-PCR assays. Taken together, Gpx1 was the target of miR-214 in PC12 cells.

### 3.5. PVT1 Knockdown Attenuated Ischemic Injury through miR-214/Gpx1 in PC12 Cells

To identify whether the PVT1/miR-214/Gpx1 signaling axis was involved in the progression of ischemic injury, rescue experiments in OGDR PC12 cells were performed. PC12 cells were transfected with the si-PVT1 along with or without miR-214 inhibitor or Gpx1 vector prior to OGDR. As shown in Figures 5(a) and 5(b), Gpx1 expression decreased by si-PVT1 was increased by the miR-214 inhibitor or Gpx1 vector. CCK-8 results discovered that PVT1 knockdown decreased PC12 cells viability, while the miR-214 inhibitor or Gpx1 vector increased cell viability (Figure 5(c)). Moreover, the expression of PCNA decreased by PVT1 knockdown was significantly elevated by miR-214 inhibition or Gpx1 promotion (Figure 5(d)). In addition, western blotting results showed that the miR-214 inhibitor or Gpx1 vector overturned the promotion effect of si-PVT1 on OGDR PC12 cell apoptosis (Figure 5(e)). Furthermore, the ROS and inflammatory cytokines in OGDR PC12 cells increased by si-PVT1 were decreased by the miR-214 inhibitor or Gpx1 vector (Figures 5(f) and 5(g)). These data demonstrated that PVT1 knockdown facilitated cell proliferation and alleviated apoptosis, ROS generation, and inflammation in ischemic stroke cells via the miR-214/Gpx1 signaling axis.

## 4. Discussion

Growing evidence has shown that lncRNAs are considered a new type of diagnostic biomarker and a promising therapeutic target for ischemic stroke. Lu et al. found that PVT1 level was upregulated in the plasma of acute ischemic stroke patients [25]. However, the functional role of PVT1 in cerebral ischemia has not been confirmed. As far as we know, PVT1 has been discovered as a tumor promoter that facilitates cell proliferation, invasion, and migration in various tumors [26–28]. This present study revealed that PVT1 was increased in OGDR-treated PC12 cells. PVT1 inhibition promoted cell proliferation and alleviated apoptosis and inflammation in OGDR PC12 cells. These findings demonstrated that PVT1 knockdown might have neuroprotective effect against OGDR-induced injury.

PVT1 was reported to be involved in several central neuronal system diseases [29, 30]. For instance, silence of PVT1 decreased the loss of neurons and inhibited the activation of astrocytes in hippocampus tissues of epileptic rats [31]. Jin et al. discovered that PVT1 promoted glioblastoma multiforme progression [8]. Moreover, it has been reported that PVT1 is involved in Parkinson's disease and Alzheimer's disease development [3]. In this current study, we displayed that PVT1 was increased in ischemic stroke, which was in line with the previous study which reported that PVT1 was highly expressed in the plasma of acute ischemic stroke [25]. Also, PVT1 knockdown attenuated cell apoptosis and inflammation in OGDR PC12 cells.

It has been reported that miRNAs modulate mRNA translation via targeting their 3′-UTR. Increasing evidence has shown the dysregulation of miRNAs in ischemic stroke, indicating the association of miRNAs with ischemic stroke. This present study demonstrated that miR-214 was validated to bind to PVT1 and was negatively modulated by PVT1. Previous research has found that reexpression of miR-214 relieves cerebral ischemic injury [32]. In line with the above studies, we found that miR-214 knockdown reversed PVT1 inhibition effect on OGDR PC12 cells. Furthermore, Gpx1 was a direct target of miR-214. Previous research has reported that Gpx1 participates in the modulation of ischemia related diseases. Similarly, we illustrated that Gpx1 is increased in ischemic stroke *in vitro*, and overexpression of Gpx1 enhanced cell apoptosis, ROS generation, and inflammation reduced by si-PVT1.

## 5. Conclusions

Here, we found that Gpx1 restoration attenuated si-PVT1 effect on OGDR induced cell apoptosis and inflammation injury, suggesting that PVT1 knockdown inhibits ischemic stroke injury via regulation of miR-214/Gpx1 axis.

## Figures and Tables

**Figure 1:** PVT1 was overexpressed in OGDR PC12 cells. (a) qRT-PCR analysis of PVT1 and (b) miR-214 mRNA level in OGDR PC12 cells. (c) Western blotting analysis of Gpx1 level in OGDR PC12 cells. ^∗∗^*p* < 0.01. Data were shown as the mean ± SD based on three independent experiments.

**Figure 2:** PVT1 knockdown attenuated ischemic injury through miR-214/Gpx1 in OGDR PC12 cells. (a) PVT1 expression was measured by qRT-PCR in si-PVT1 PC12 cells. (b) CCK-8 analysis of si-PVT1 effect on PC12 cell viability. (c) qRT-PCR analysis of si-PVT1 role on PCNA expression. (d) Western blotting analysis of si-PVT1 effect on Bcl-2, Bax, and cleaved-caspase-3 levels in PC12 cells. (e) ELISA assay analysis of the effect of si-PVT1 on the productions of ROS and (f) IL-6, IL-1*β*, and TNF-*α* in OGDR PC12 cells. ^∗∗^*p* < 0.01 and^∗∗∗^*p* < 0.001; ^#^*p* < 0.05 and^##^*p* < 0.01. Data were shown as the mean ± SD based on three independent experiments.

**Figure 3:** PVT1 functions as a ceRNA of miR-214 in PC12 cells. (a) The binding sites of PVT1 and miR-214, as shown by Starbase. (b) Detection of miR-214 expression in PC12 cells. (c) Measurement of the luciferase activity of PVT1. (d) Measurement of PVT1 or miR-214 expression in Ago2, IgG, and Input groups. (e) Detection of PVT1 expression by qRT-PCR. (f) Observation of PVT1 effect on miR-214 expression by qRT-PCR. ^∗∗^*p* < 0.01 and^∗∗∗^*p* < 0.001. Data were shown as the mean ± SD based on three independent experiments.

**Figure 4:** miR-214 directly targeted Gpx1 in PC12 cells. (a) The binding sites of Gpx1 and miR-214, as shown by Starbase. (b) Measurement of the luciferase activity of Gpx1. (c) qRT-PCR analysis of Gpx1 mRNA expression. (d) Detection of Gpx1 protein level by western blotting. ^∗∗^*p* < 0.01. Data were shown as the mean ± SD based on three independent experiments.

**Figure 5:** PVT1 knockdown attenuated ischemic injury through miR-214/Gpx1 in PC12 cells. PC12 OGDR cells were treated with si-PVT1, combined with miR-214 inhibitor or pcDNA-Gpx1. (a) Measurement of the mRNA expression or (b) protein level of Gpx1. (c) CCK-8 analysis of the cell viability. (d) QRT-PCR analysis of PCNA expression. (e) Western blotting analysis of Bcl-2, Bax, and cleaved-caspase-3 levels. (f) ELISA assay analysis of the levels of ROS and (g) IL-6, IL-1*β*, and TNF-*α*, respectively. ^∗∗^*p* < 0.01;  ^#^*p* < 0.05;  ^&^*p* < 0.05. Data were shown as the mean ± SD based on three independent experiments.

## Data Availability

The datasets used and/or analyzed during the present study are available from the corresponding author on reasonable request.
